This article has been retracted.

# miR-211 suppresses hepatocellular carcinoma by downregulating SATB2

**DOI:** 10.18632/oncotarget.3265

**Published:** 2015-03-25

**Authors:** Guixing Jiang, Yunfu Cui, Xin Yu, Zhengrong Wu, Guoping Ding, Liping Cao

**Affiliations:** ^1^ Department of Hepatopancreatobiliary Surgery, Sir Run Run Shaw Hospital, School of Medicine, Zhejiang University, Hangzhou, China; ^2^ Department of Hepatopancreatobiliary Surgery, Second Affiliated Hospital of Harbin Medical University, Harbin, China; ^3^ Department of Biochemistry and Molecular Biology, Institute of Basic Medical Sciences, Chinese Academy of Medical Sciences, Beijing, China

**Keywords:** hepatocellular carcinoma, microRNAs, miR-211, SATB2

## Abstract

Dysregulation of microRNAs (miRs) is involved in carcinogenesis. Deregulation of miR-211 has recently been observed in many tumors, but its function in hepatocellular carcinoma (HCC) is still unknown. Here we found that miR-211 was decreased in HCC cancer tissues compared with adjacent normal tissues. We also found that overexpression of miR-211 repressed proliferation and invasion in HepG2 and SMMC7721 cells. Luciferase reporter assays and western blot indicated that special AT-rich sequence-binding protein-2 (SATB2), is a direct target of miR-211. The expression of SATB2 was upregulated in HCC cancer tissues and cell lines and miR-211 levels inversely correlated with SATB2 levels in HCC. Importantly, SATB2 rescued the miR-211-mediated inhibition of cell invasion and proliferation. Finally, reintroduction of miR-211 repressed tumor formation of HCC in xenograft mice. This study provides insights into molecular mechanisms that miR-211 contributed to HCC.

## INTRODUCTION

Hepatocellular carcinoma (HCC) is the sixth most prevalent cancer and the third most frequent cause of cancer mortality worldwide, leading to more than 600,000 deaths each year [1, 2]. HCC is especially common in China, with the mortality rate the second highest [3]. In China, more than 110 000 people die from liver cancer each year, causing 45% of the liver cancer death in the world [3]. Despite therapeutic advances, the 5-year survival rate of HCC is still below 5% [4–6]. HCC is the result of a multistep process, which involves the accumulation of several structural and genomic alterations [7, 8]. Hence, it is urgent to develop novel strategies for the early diagnosis, prediction of the prognosis and therapeutic target of patients with HCC.

MiRNAs are a group of endogenous, small, non-coding RNAs that negatively regulate gene expression via binding to the 3′untranslated region (3′UTR) of mRNA, leading to repress post-transcripional translation or the degradation of the target mRNA [9–12]. Increasing researches have indicated that deregulation of miRNAs plays large roles in the initiation and progression of many cancers such as breast cancer, gastric cancer, lung cancer, and bladder cancer [13–17]. Through regulating various target mRNAs gene, miRNAs are involved in many biological processes including cell proliferation, apoptosis, invasion, migration, differentiation, angiogenesis and immune response, metabolism, and so on [18–21]. Therefore, better knowledge of changes in miRNA gene expression during live carcinogenesis and metastasis may provide new avenues for HCC diagnostic and treatment regiments [22–26].

In this study, we aimed to determine the expression and function of miR-211 in HCC and investigate the molecular mechanism of miR-211 in the initiation and progression of HCC.

## RESULT

### MiR-211 is downregulated in HCC cell lines and tissues

The decrease of miR-211 was found in 33 of 40 HCC tissues compared with the corresponding non-tumor tissues (Figure 1A). As shown in Figure 1B, the expression of miR-211 in HCC tissues was lower than in adjacent tissues (Figure 1B, *p* < 0.001). Moreover, tissues from lymph node metastases also expressed lower levels of miR-211 compared with primary HCC tissues and the adjacent normal tissue (Figure 1C). As shown in Figure 1D, the expression of miR-211 was significantly down-regulated in four cell lines (MHCC-97H, QGY-7703, SMMC7721 and HepG2) compared with one liver adenocarcinoma cell line, SK-Hep-1, and two adjacent non-neoplastic tissues.

**Figure 1:** miR-211 is downregulated in HCC cell lines and tissues **(A)** qRT-PCR analysis of miR-211 expression in 40 pairs HCC tissues and their corresponding no tumor tissues. The expression of miR-211 was normalized to U6 snRNA. **(B)** The expression of miR-211 in HCC tissues was significant lower than in adjacent tissues. **(C)** The expression of miR-211 in 10 pairs lymph node metastases, HCC tissues and their corresponding to no tumor tissues. **(D)** Expression levels of miR-211 in four cell lines (MHCC-97H, QGY-7703, SMMC7721 and HepG2) compared with one liver adenocarcinoma cell line, SK-Hep-1, and two adjacent nonneoplastic tissues were detected using qRT-PCR analysis. *p < 0.05 and ***p < 0.001.

### Upregulation of miR-211 inhibits cell proliferation

To study the role of miR-211 in HCC development, SMMC7721 and HepG2 were transfected with miR-211 mimics or inhibitor with high transfection efficiency (Figure 2A and 2B). Down expression of miR-211 inhibited the growth rate of HCC cells compared with control cells in both SMMC7721 and HepG2 cells (Figure 2C and 2D). Conversely, miR-211 mimics promoted the proliferation of the HepG2 cells in both SMMC7721 and HepG2 cells (Figure 2C and 2D).

**Figure 2:** Upregulation of miR-211 inhibits cell proliferation **(A)** miR-211 mimics can enhance the expression of miR-211 and miR-211 inhibitor can repress the expression of miR-211 in the HepG2 cells. **(B)** miR-211 mimics can enhance the expression of miR-211 and miR-211 inhibitor can repress the expression of miR-211 in the SMMC7721 cells. **(C)** CCK-8 proliferation assay showed that overexpression of miR-211 significantly inhibited the growth rate of cells compared with control cells in both and HepG2cells. Conversely, miR-211 inhibitor significantly promoted the proliferation of the HepG2 cells. **(D)** CCK-8 proliferation assay showed that overexpression of miR-211 significantly inhibited the growth rate of cells compared with control cells in both and SMMC7721 cells. Conversely, miR-211 inhibitor significantly promoted the proliferation of the SMMC7721 cells. *p < 0.05, **p < 0.01, and ***p < 0.001.

### Upregulation of mir-211 inhibits cell invasion

Overexpression of miR-211 can promote the invasion of HepG2 cells and SMMC7721 compared with the control whereas miR-211 inhibitor inhibited cell invasion (Figure 3A and 3B). The relative invasive cells of each group were shown in the right.

**Figure 3:** Upregulation of miR-211 inhibits cell invasion **(A)** Upexpression of miR-211 can significantly promoted the HepG2 cells invasion whereas miR-211 inhibitor inhibitedHepG2cell invasion. The relative invasive cells of each group have been shown in the right. **(B)** Upexpression of miR-211 can significantly promoted the SMMC7721 cells invasion whereas miR-211 inhibitor inhibited SMMC7721 cell invasion. The relative invasive cells of each group have been shown in the right. ***p < 0.001.

### stab2 is a direct target of mir-211

Using bioinformatics analysis, we found that 3′-UTR of STAB2 contained a conserved putative target site for miR-211 (Figure 4A). Therefore, the 3′-UTR of human STAB2 was amplified and inserted into downstream of the luciferase gene in the pGL3-control vector. As shown in Figure 4B, miR-211 mimics repressed the luciferase activity. Mutation of miR-211 binding site from the STAB2 3′-UTR largely abolished the effects of miR-211 mimics. Meanwhile, miR-211 repressed the mRNA expression of STAB2. In addition, Western blot analysis also showed that ectopic expression of miR-211 markedly suppressed STAB2 expression in HepG2 cell line (Figure 4C and 4D).

**Figure 4:** STAB2 is a direct target of miR-211 **(A)** Predicted miR-211 target sequence in the 3′UTR of STAB2 and mutant containing 8 altered nucleotides in the 3′UTR of STAB2. **(B)** The analysis of the relative luciferase activities of STAB2-WT, STAB2-MUT in the HepG2 cells. **(C)** qRT-PCR analysis of STAB2 mRNA expression in the HepG2cellscells after treatment with miRNA mimics or scramble or no transfection. The expression of STAB2 was normalized to GAPDH. **(D)** Western blot analysis of STAB2 expression in the HepG2 cells transfected with miR-564 mimics or scramble or no transfection. GAPDH was also detected as a loading control. ***p < 0.001.

### miR-211 regulated cell proliferation and invasion through inhibiting SATB2

The SATB2 expression vector pcDNA-SATB2 was used to restore SATB2 expression (Figure 5A and 5B). Overexpression of SATB2 promoted the HepG2 cells proliferation and invasion (Figure 5C and 5D). As expected, the ectopic expression of SATB2rescued the miR-211-mediated inhibition of cell proliferation and migration in HepG2 cells (Figure 5C and 5D).

**Figure 5:** miR-211 regulated cell proliferation and invasion through inhibiting SATB2 **(A)** The protein expression of SATB2 was detected using western blot in HepG2 cells. GAPDH was also detected as a loading control. **(B)** The mRNA expression of SATB2 was detected using qRT-PCR in HepG2 cells. The expression of STAB2 was normalized to GAPDH. **(C)** Cell proliferation was determined by CCK-8 assay. The ectopic expression of SATB2 rescued the miR-211-mediated inhibition of cell proliferation in HepG2 cells. **(D)** The ectopic expression of SATB2 rescued themiR-211-mediated inhibition of cell invasion in HepG2 cells. *p < 0.05, and **p < 0.01, ***p < 0.001.

### STAB2 was inversely expressed with miR-211 in HCC patients

As shown in Figure 6A and 6B, STAB2 was up-regulated in four cell lines (MHCC-97H, QGY-7703, SMMC7721 and HepG2) compared with one liver adenocarcinoma cell line, SK-Hep-1, and two adjacent tissues. To further validate our findings, the levels of STAB2 were measured in 20 human primary HCC and pair-matched peri-tumoral tissues. As shown in Figure 6C, the expression of STAB2in HCC tissues was lower than in adjacent tissues (Figure 1C, *p* < 0.001). The increase of STAB2 was found in 19 of 20 HCC tissues compared with the corresponding non-tumor tissues (Figure 6D). Comparison of miR-211 levels and levels corresponding to STAB2 in HCC exhibited inverse correlation between STAB2 and miR-211 (*r*^2^ = 0.426, *p* = 0.0018) (Figure 6E).

**Figure 6:** STAB2 was inversely expressed with miR-211 in HCC patients **(A)** Expression levels of STAB2 in four cell lines (MHCC-97H, QGY-7703, SMMC7721 and HepG2) compared with one liver adenocarcinoma cell line, SK-Hep-1, and two adjacent nonneoplastic tissues were detected using qRT-PCR analysis. **(B)** The protein expression levels of STAB2 in four cell lines (MHCC-97H, QGY-7703, SMMC7721 and HepG2) compared with one liver adenocarcinoma cell line were detected using western blot. **(C)** The expression of STAB2in HCC tissues was significant lower than in adjacent tissues. **(D)** The increase of STAB2 was found in 19 of 20 compared with the corresponding non-tumor tissues. **(E)** Comparison of miR-211 levels and levels corresponding to STAB2 in HCC exhibited significantly inverse correlation between STAB2 and miR-211 (*r*2 = 0.426, *p* = 0.0018). ***p < 0.001.

### miR-211 inhibited the growth of HepG2-engrafted tumors

MiR-211 mimic injection repressed the growth of HepG2-engrafted tumors compared to scrambled oligonucleotides-treated tumors (Figure 7A). In agreement with the tumor growth curve, the volumes and weights of tumors treated by miR-211 mimics were also lower than scrambled mimics-treated tumors (Figure 7B and 7C). Western blot analysis in randomly selected xenograft mouse tumors showed that miR-211 mimics-injecting tumors expressed lower levels of STAB2 than scramble controls (Figure 7E). Moreover, Ki-67 was lower in the miR-211 mimics-injecting tumors compared to the scrambled mimics-treated tumors (Figure 7D).

**Figure 7:** miR-211 repressed the growth of HepG2-engrafted tumors **(A)** Representative tumors were photographed at 15 days after the first treatment with miR-211 mimic or scramble. **(B)** Tumor weight averages between scrambled and miR-211 mimics-treated mice groups at the end of the experiment (day 25). **(C)** Graph representing tumor volumes at the indicated days during the experiment for the two groups: scrambled mimics, miR-211 mimics. **(D)** Injection of miR-211 reduced Ki-67 protein expression in HepG2 xenograft tumors. **(E)** Injection of miR-211 reduced STAB2 protein levels in HepG2 xenograft tumors. Represented are 2 tumors from each group. ***p < 0.001.

## DISCUSSION

The important role of deregulated miRNAs in cancer has been proved by many researches [18, 19, 28–30]. Our study showed that miR-211 expression was downregulated in HCC cells and HCC tissues. Furthermore, ectopic expression of miR-211 repressed the proliferation and invasion of HCC cells. As for the mechanism, our results indicated that miR-211 directly targeted SATB2 to inhibit cell proliferation and invasion in HCC cells. Importantly, SATB2 rescued the miR-211-mediated inhibition of cell invasion and proliferation. Moreover, our investigation for the expression of SATB2 and miR-211 in 20HCC patients indicated that there was an inverse correlation between miR-211 and SATB2 levels. These findings suggest that miR-211 may play an important role in promoting carcinogenesis of HCC.

Researchers have illustrated that miR-211 is abnormally expressed in various tumors and directly involves in human cancer processes, such as cell proliferation, migration and metastasis [31–36]. MiR-211 was upregulated in oral carcinoma and higher miR-211 expression was associated with nodal metastasis, vascular invasion, and poor prognosis of oral carcinoma [32]. Moreover, enforced miR-211 expression increased the proliferation, migration, and anchorage-independent colony formation of oral carcinoma cells. Furthermore, enforced expression of miR-211 promoted tumor cell growth at least in part by down-regulating the CHD5 tumor suppressor [31]. On the other hand, another study showed that miR-211 was a suppressor of melanoma invasion during human melanoma progression [34, 37, 38]. To our knowledge, the role and mechanism of miR-211 in HCC have not been completely understood. Our results indicated that miR-211 was down-regulated in HCC tissues compared with adjacent non-neoplastic tissues. Moreover, tissues from lymph node metastases expressed lower levels of miR-211 compared with primary HCC tissues and the adjacent normal tissue, indicating an inverse relationship between miR-211 and the metastatic status of HCC. Furthermore, over-expression of miR-211 could repress HCC cell proliferation and invasion. These results suggested that miR-211 might act as a tumor suppressor whose down-regulation contributed to the progression and metastasis of HCC.

Integrating bioinformatics and experimental assays, we identified SATB2 as a direct downstream target of miR-211 in HCC cells. Complementary sequence of miR-211 was identified in the 3′UTR of SATB2 mRNA. Overexpression of miR-211 reduced SATB2 both mRNA and protein levels in HCC cells. Moreover, miR-211 decreased the luciferase reporter activity of wild-type 3′UTR but not mutant 3′UTR of SATB2. Human special AT-rich sequence-binding protein-2 (SATB2) is a novel AT-rich DNA binding protein, which is involved in regulating gene expression through altering chromatin structure [39–42]. Previous studies have shown that SATB2 directly interacts with the activity of transcription factors which regulate cortical neurons differentiation and craniofacial development [43, 44]. It has been demonstrated that the expression of SATB2 was lower in primary colorectal cancer (CRC) [45]. Furthermore, down-regulated expression of SATB2 was associated with metastasis and poor prognosis in CRC [45]. Another study has reported that SATB2 was associated with increasing tumor grade and poorer overall survival in breast cancer [46]. However, the expression and mechanism of SATB2 in HCC remain unknown. In our study, SATB2 expression is up-regulated in HCC tissues compared with adjacent pair-matched non-tumor tissues. The expression of SATB2 is also increased in the HCC cells. Moreover, SATB2 rescued the miR-211-mediated inhibition of cell invasion and proliferation and there was an inverse correlation between miR-211 and SATB2 levels in HCC tissues. These results demonstrate thatSATB2 is a functional target gene of miR-211 in HCC.

To our knowledge, there is no study on miR-211 and HCC tumorigenicity in a xenograft model. In our research, the tumor-suppressive role of miR-211 *in vivo* was treated through direct miRNA mimics injection. Our result proved that miR-211 significantly inhibited the growth of HCC cells. Further western blot analysis demonstrated the negative regulation of miR-211 to SATB2. These results suggest that miR-211 might be a potential therapeutic choice in HCC.

In conclusion, we identified that miR-211 acted a tumor suppressive miRNA in HCC tumorigenesis and progression. Given that reintroduction of miR-211 inhibited tumor formation in xenograft model, this mature miRNA could serve as a potential therapeutic strategy for HCC. Our findings are encouraging and suggest that this miRNA could be targeted for the development of novel treatment for HCC in the futur

## MATERIALS AND METHODS

### Patients and samples

Tumor tissues from HCC patients and paired adjacent non-cancerous specimens were obtained from patients undergoing surgery at Sir Run Run Shaw Hospital. None of these patients had received local or systemic anti-cancer treatment before surgery. The patient information is summarized in Supplementary Table S1. All tissues were collected immediately during surgery and stored at −80°C until the RNA and protein were later extracted. The studies were approved by the ethics committee of Sir Run Run Shaw Hospital.

### Cell lines and culture

Cell lines derived from human hepatocellular carcinoma (MHCC-97H, QGY-7703, SMMC7721, HepG2) and liver adenocarcinoma (SK-Hep-1) were incubated and cultured in Dulbecco's modified Eagle's medium (DMEM, Hyclone, Logan, UT, USA), which was also supplemented with 10% fetal bovine serum (FBS, Hyclone, Thermo Fisher Scientific, Mordialloc, Victoria, Australia).

### RNA extraction and quantitative real-time PCR

Total RNA was extracted from cell lines or frozen tissues using Qiazol reagent and miRNeasy mini kit (Qiagen, Valencia, CA, and USA). The qRT–PCR reactions were performed using iQSYBR Green super mix (Bio-Rad, Hercules, CA, USA). To determine the threshold cycle (Ct) when exponential amplification of the PCR products began, an iQ-5 (Bio-Rad) was used to monitor the PCR in real-time. The average Ct, from triplicate assays, was used for further calculations. Primers are listed in Supplementary Table S2. Relative expression levels were normalized to control. The endogenous U6 snRNA or GAPDH was chosen as the internal control.

### Oligonucleotides and transfection

MiR-211 mimics/inhibitors and negative control molecules (scramble control mimic and inhibitor) and pcDNA-SATB2 were purchased from Dharmacon (Austin, TX, USA). Cell transfection was performed using DharmFECT1 (Dharmacon) until a final concentration of 20 nM. Medium was changed after 6 h. After transfected and cultured for 48 h, cells were collected for Western blot and qRT-PCR analyses.

### Cell proliferation assay

Cell Counting Kit (CCK-8) assay was used for cell proliferation analysis. Cells were cultured in 10% CCK-8 (DOJINDO) diluted in normal culture media at 37°C. When visual color conversion appeared, quantification was carried out on a micro titer plate reader (Spectra Rainbow; Tecan).

### Cell invasion assay

Invasion assays were performed in triplicate using Transwell invasion chambers coated with Matrigel (50 μl per filter) (BD Biosciences, Franklin Lakes, NJ, USA) in accordance to the manufacturer's protocol. After being cultured for 48 h, cells were transferred on the top of Matrigel-coated invasion chambers in a 1% fetal calf serum DMEM/F12 (2 × 10^4^ cells/well). The lower chambers were added with DMEM/F12 containing 10% fetal calf serum. Cells were incubated for 24 h at 37°C in an atmosphere containing 5% CO2. Subsequently, invaded cells on the lower surface were stained with crystal violet stain and counted under a light microscope.

### Western blot

Western blots were performed as previously described [27]. Proteins were resolved with10% SDS-PAGE gel, subsequently transferred to the nitrocellulose membrane. Then the membranes were, blocked in 5% non-fat dry milk in Tris-buffered saline (pH 7.4) containing 0.05% Tween-20 and blotted with a rabbit polyclonal antibody against SATB2 and GAPDH (1:1,000; Santa Cruz Biotechnology, Inc., Santa Cruz, CA, USA) and goat anti-rabbit IgG. GAPDH were chosen as a loading control. Protein bands were detected by chemilumine scenceusing the ECL system (Vigorous Biotech, Beijing, China).

### Luciferase reporter assays

Cells in 24-well plates (50% confluency) were co-transfected with miR-211 mimic (20 nM) and STAB2 3′UTR Reporter (200 ng). Luciferase activity was detected 24 h later using the Dual-Glo luciferase assay system (Promega, Fitchburg, WI, USA) according to the manufacture's protocol.

### *In vivo* studies

Animal xenograft model studies were carried out according to institutional guidelines; HepG2 cells (3 × 10^6^) were injected subcutaneously into the posterior flanks of 6-week female nude mice, with a frequency of every 3 days for a total of six times. On the 10th day after injection, tumor diameters were measured every 3 days. On the 25th day after injection, mice were killed. Tumors were collected and weighted after necropsy. Tumor volume was calculated as length × width 2 × ½ mm^3^. When tumor size reached 50 mm^3^, miRNA mimics diluted in Lipofectamine 2000 (Invitrogen) solution (100 nmol mimics in 100 μl total volume) were injected into the tumors.

### Statistics

Data were presented as the mean ± standard deviation (SD) from three separate experiments. When two groups were compared, the differences between groups were analyzed using Student's *t*-test and when more than two groups were compared, a one-way analysis of variance (ANOVA) was used. The differences between groups of metastasis *in vivo* were analyzed using the χ2 test. All statistical analyses were performed with SPSS 16.0 (SPSS Inc., USA). The difference was considered statistically significant at *p* < 0.05.

## SUPPLEMENTARY TABLES


